# Depletion of Amoxicillin Residue in Edible Tissue of Broiler Chicken by Different Cooking Methods

**DOI:** 10.1155/2022/7812441

**Published:** 2022-08-24

**Authors:** Aynalem Lakew, Negussie Megersa, Bhagwan S. Chandravanshi

**Affiliations:** ^1^Department of Chemistry, College of Natural and Computation Sciences, Addis Ababa University, P.O. Box 1176, Addis Ababa, Ethiopia; ^2^Ethiopian Public Health Institute, P. O. Box 1242/5654, Addis Ababa, Ethiopia

## Abstract

A new simple isocratic, RP-HPLC method, was developed and validated to estimate amoxicillin (Amox) residue depletion caused by different cooking methods in broiler chicken tissue. The limit of detection (LOD) and the limit of quantitation (LOQ) were 1.32 and 4.00 *µ*g mL^−1^, respectively. The calibration plot was linear over the concentration range of 0.05–250 *µ*g mL^−1^, and the relative standard deviation (RSD) values were less than 8%. The effects of various cooking methods (boiling, pan-frying, and microwaving) on residues of Amox were conducted under different combinations of temperature and time. Moreover, the heat stability of Amox standard solutions under boiling water and cooking oil at 100°C was investigated. Amox remained stable for 5–15 min in boiling water, the concentration was significantly reduced in the range of 70–87%, and additional new peaks of the degraded compounds appeared at 30–45 min. In pan-frying, the residue remained stable for 15 min at 100°C and then depleted to 81–92% after 30–45 min. Due to dehydration, the residue concentration showed an increment from 101 to 112% at 150°C. The total decomposition of Amox was observed at 200°C, 30–45 min due to high temperature and long-time effects. In microwave cooking using 500 W, 0.5–2 min, the depletion was insignificant. This study shows that sufficient cooking temperature and time can have a significant effect on the depletion of Amox residues.

## 1. Introduction

Antimicrobial resistance and antibiotic residues are considered a global public health concern today, and it affects all countries [1]; however, its burden on low-income countries, like Ethiopia, is relatively high [2]. The antimicrobial use was highest in chickens at 138 doses/1000 animal days in low- and middle-income countries [3]. Antibiotics in poultry production are a key contributor to antimicrobial resistance (AMR) risk because the edible parts of treated animals or the byproducts may contain the residue of drugs [4]. In poultry productions, proper antibiotic use and good veterinary practices prevent bacterial infections, cure diseases, enhance growth and feed efficiency, and produce healthy and fresh edible chicken products [5]. However, the overuse of these antibiotics, improper treatment, and insufficient withdrawal time may lead to the presence of antibiotic residues in edible tissues intended for human consumption which also resulted in health risks to the consumer [6]. The possible human health hazard caused by antibiotic residues in poultry meat includes allergic reactions, sensitivity to drugs, imbalance of intestinal microbiota, a mutation in cells, and bacterial resistance to antibiotics [7].

Most reported information regarding antibiotic residues in chickens is related to their concentrations before cooking [8, 9]. However, most chicken tissue parts are not consumed raw, and different methods such as boiling, roasting, barbequing, steaming, frying, or microwaving are used for cooking the chicken meat [10, 11]. Cooking results in denaturation of protein, elevation of temperature, and change of the existing concentration of chicken tissue components including antibiotic residues, pH, chemical nature, and solubility. Heat treatments can cause drug residue loss through evaporation or thermal degradation [4]. The effects of heat treatment on residues of antimicrobials are dependent on the type of cooking in addition to other processes like fermentation, storage time, and conditions that also have considerable impacts on the depletion of drug residues [12]. Data on the effect of heat treatment on the normal cooking procedure is essential to provide a more precise estimate of the concentration of parent drug residues and any breakdown products that the users may be exposed to [4].

The heat stabilities of antibiotics have been studied based on microbiological screening assays (antimicrobial activity) or by chromatographic analysis (change in concentration after heat treatments) [13]. Few studies have reported on the impact of domestic cooking practices and heat stability of antibiotics in chicken tissue using both microbiological and chemical analyses [14]. The effects of cooking on the depletion of antibiotic residues in fortified and incurred chicken tissues were done for enrofloxacin [12], oxytetracycline [15], gentamicin, oxytetracycline, and tilmicosin [15]. Since the literature information about the effects of cooking on drug residues is still insufficient, the risk to the consumer from dietary exposure to these residues is not well known [16].

In several African countries, tetracyclines are highly predominant antibiotics and represent 41% of all antibiotic contaminants in chicken samples (meat and liver), followed by *β*-lactams at 18% [17]. Amoxicillin is used in a wide range of livestock species including chicken and can be administrated either orally or by injection for the treatment of susceptible infections of the alimentary and respiratory tracts [18]. In Ethiopia, few researchers conducted a cross-sectional study using bacteriological methods to estimate Amox residues in animal-derived foods, and they have reported the drug concentration was exceeded the World Health Organization (WHO) maximum residue levels. Recently, 51.6% resistance to amoxicillin was reported in a hospital-based cross-sectional survey by Ejerssa and coworkers [19]. Similarly, other literature reports have also indicated that 9.5–19% of *Salmonella* isolates were resistant to amoxicillin and other antimicrobials on food items of animal origin [20, 21].

However, there is limited information on the effects of cooking on amoxicillin residues in chicken muscles, and this creates a scientific gap of knowledge that needs to be addressed. Thus, this study investigates the effects of household cooking activities such as boiling, pan-frying, and microwave cooking on Amox residues in tissues of broiler chickens using liquid chromatographic analysis.

## 2. Materials and Methods

### 2.1. Chemicals and Reagents

All the reagents and chemicals used in this study were of analytical grade. Standard reference amoxicillin (99% purity) Sigma-Aldrich Chemical Company (St. Louis, USA) was kindly provided by the Ethiopian Food and Drug Administration (EFDA). The chemical and structural formula of amoxicillin is illustrated in Figure 1. Both methanol and acetonitrile (>99%) were HPLC grade solvents, obtained from Merck (Germany). Disodium hydrogen phosphate (>99%), orthophosphoric acid (>85%), and sodium hydroxide (>85%) were purchased from Sigma-Aldrich (USA). The blank chicken sample, without any antibiotics including amoxicillin, is referred to as tissue performance negative concentration CHARM II kit, lot TPNC-053, was a kind donation of the Ethiopian Public Health Institute (EPHI) and Water Still, 4 LPH, double distilled, 240 VAC, 50/60 Hz from Stuart Aquatron (USA) used to purify the water throughout the experiment.

### 2.2. Materials and Equipment

Filtration of the standards and samples was done by syringe membrane filters (0.45 *μ*m Millex-HN; Millipore; Bedford, MA, USA). Vortex mixer (Vortex-Genie 2; Scientific Industries Inc., Bohemia, New York, USA) and ultrasonic machine (B5510J-DTH; Branson, Danbury, CT) were used for homogenization. Centrifuge, AX-320 (Tomy Seiko Co., Tokyo, Japan), was used to separate the organic layer of solutions. The pH meter (Hanna Instruments Inc., Cluj-Napoca Jud, Cluj, Romania) was used to measure the pH of the solutions. Mobile phase solvents were purified using vacuum filtration assembly (Millipore filter cellulose nitrate gridded with 0.22 *μ* size and 47 mm diameter, Sigma-Aldrich (USA)). Kitchen utensils, stainless steel laboratory knife, frying pan, and Pyrex beaker were used in sample preparation and cooking experiments. The temperature achieved during each cooking procedure was monitored using a 5″ Analog Pocket Test Chef Thermometer with 50 to 550 (°F) ± 5°F accuracy in Stainless Steel Stem (Trump, China). LMV1831BD-Over-the-Range Microwave Oven, 1000 Watts (LG, USA), was used to cook the chicken tissues. R2B CLR Cutter Mixer Clear Polycarbonate Batch Bowl (Robot Coupe USA) was used to blend the chicken meat.

### 2.3. Instruments and Chromatographic Separation

The concentrations of Amox residue in the raw and cooked chicken were determined by LC (Shimadzu prominence LC-20AD system, Kyoto, Japan). The instrument is equipped with quaternary pumps, a dual wavelength UV detector, a column oven, and an automatic sample injector. The chromatographic separation was performed with reversed phase and isocratic elution on Hypersil BDS-C18 (3 *μ*m, 100 mm × 4 mm) (Phenomenex, USA). The mobile phase for LC analysis consisted of a combination of 0.05 M Na_2_HPO_4_, acetonitrile, and methanol (70 : 10 : 20 v/v/v) at pH 8. The injected volume was 20 *μ*L with a flow rate of 1 mL min^−1^ at ambient temperature, and the compounds were detected at 230 nm.

### 2.4. Preparation of Buffer and Standard Solutions

The stock standard solution (1000 *μ*g mL^−1^) was prepared by weighing 10 mg of Amox in a 10 mL volumetric flask and dissolving in 1 : 1 methanol : deionized water (v/v) and kept in amber colored containers for one month at −5°C. For recovery experiments, working standard solutions of (10, 100, and 200 *µ*g mL^−1^) were prepared fresh daily by serial dilution of the Amox stock solution to avoid any possible degradation caused by prolonged storage. Phosphate buffer (0.05 M pH 8) was prepared by weighing 7.097 g of disodium hydrogen phosphate (Na_2_HPO_4_.12H_2_O) in a 1000 mL volumetric flask containing 900 mL deionized water and dissolved, and then the final volume was filled to the mark. The final desired pH was adjusted using orthophosphosphoric acid or NaOH, and all solutions were filtered through a 0.45 *μ*m membrane filter.

### 2.5. Sample Preparation

One kilogram of slaughtered and market-ready broiler chicken was bought from the local market of Addis Ababa, Ethiopia. All adhering connective tissues were removed from the muscles, deboned, each large individual muscle separated, and the meat was then cut into chunks of 4–8 cm sizes and washed with potable water several times, rinsed with distilled water, put through a sieve to dry the water, ground in a Bowl Cutter Mixer, and kept at −20°C.

### 2.6. Statistical Analysis

The data obtained for each parameter was subjected to statistical analysis using Fisher's statistical test in Excel for analysis of the variance (ANOVA). The parameters for the validation and calibration line settings were performed using Microsoft Office Excel 2010 software. All the measurements were carried out in triplicate.

### 2.7. Cooking Processes

#### 2.7.1. Stability of Amox Standards in Boiling Water

One milliliter of 1000 *µ*g mL^−1^ Amox standard solution was added into each of the six Pyrex beakers containing 9 mL of boiled water (total volume was 10 mL) at 100°C to the final concentration of 100 *µ*g mL^−1^. The solution was boiled for a specified time of 5, 15, 30, and 45 min, and 1 mL sample was taken by a 1000 *µ*L micropipette. To control preconcentration and reach out to a 100 *µ*g mL^−1^ solution of Amox, the observed volume loss of water caused by evaporation was recompensated in the beaker by the addition of boiled water before sampling in each time interval. The HPLC analysis was performed directly on the aqueous samples by filtering with syringe membrane filters, the peak area was utilized as the instrumental response for data acquisition, and processing accomplished with the LC solution software.

#### 2.7.2. Stability of Amox Standards in Cooking Oil

One milliliter of 500 *µ*g mL^−1^ standard solution of Amox was added to four 10 mL stainless steel metal centrifuge tubes containing 5 g sunflower oil. The tubes were vortex-mixed and placed in a heating module at 100°C for 30 min, removed, and allowed to cool. The sample was dissolved in 2 mL isopropanol and extracted with 2 mL acetonitrile. The resulting solution was mixed with a vortex, centrifuged at 3800 rpm for 5 min, and the supernatant was evaporated to near dryness with a stream of nitrogen. The concentrated Amox residue was re-dissolved with 2 mL MeOH and analyzed by LC.

It should be noted that we have studied the stability of Amox standards in cooking oil without adding a chicken sample. Furthermore, Amox is soluble in water (3.43 g L^−1^), slightly soluble in ethanol (96%), and practically insoluble in fatty oils [22]. Isopropanol, a polar protic solvent, was used to dissolve the oil sample and facilitate the formation of emulsion to dissolve Amox, while acetonitrile was used to extract the Amox.

#### 2.7.3. Boiling Process for Chicken Tissues

Boiling is a simple and widely used household cooking method for chicken meat in water at the boiling point of 100°C [11]. For this experiment, distilled water (500 mL) was preheated to 97–100°C in Pyrex beakers and 10 g spiked tissue samples with 5 mL 100 *µ*g mL^−1^ Amox were immersed and cooked for a specified periods of 5, 15, 30, and 45 min. The surrounding fluids (1 mL) were sampled using a 1000 *µ*L micropipette from boiled water, and 2 g of the boiled tissue sample was taken separately from the boiling water. To control preconcentration, the observed volume loss of water caused by evaporation was recompensed in a beaker with the addition of boiled water prior to sampling in each time interval. Internal muscle temperatures (°C) of the cooked samples were measured by striking the sensor probe of the thermometer into the center of the chicken meat during the cooking process. The internal temperatures were measured during cooking, and mean values were less than 80°C throughout the boiling period. The collected samples were allowed to cool to room temperature, and 10 mL acetonitrile was added to extract the residue, shaken well for 1 min, sonicated, and centrifuged at 3800 rpm for 5 min. The resulting supernatant was evaporated using a nitrogen stream and the dried sample was redissolved with 2 mL MeOH and injected into the LC.

#### 2.7.4. Pan-Frying Process for Chicken Tissues

Frying (pan-frying) is a rapid food preparation technique and the most common ordinary cooking method in which food is submerged in hot fat or cooking oil. Frying in an open (uncovered) pan promotes physical and chemical changes in the foods and leads to unique sensory properties of color, flavor, texture, and palatability [11]. To study the effect of frying in Amox residue, on the open frying pan, one tablespoon of sunflower oil was placed and heated to a temperature of 100, 150, and 200°C, and 10 g of spiked chicken tissue (100 mg L^−1^) was placed on the oil once it had reached the desired temperature, and samples were cooked. Samples were taken between 5, 15, 30, and 45 min. During this frying process, meat was stirred well with a glass rod to keep the sample homogeneous. The collected samples were cooled to room temperature and extracted as described in Section 2.8.

#### 2.7.5. Microwave Cooking for Chicken Tissues

Microwave cooking is a more recent cooking method, widely applied to reheat and cook meals. Microwave ovens work by producing electromagnetic waves via an electron tube called a magnetron contained inside the oven. The microwaves are absorbed by the food, and the waves cause the vibration of water molecules in the food, generating heat which is then transmitted throughout the food by thermal conduction. One of the major problems associated with microwave heating is uneven temperature distribution. This can result in cold spots, which may pose cause health problems for consumers with respect to the survival of bacteria in the cold spot of the meat [23].

The spiked 5 g samples were placed into plastic tubes, and the plastic cover of each tray was perforated to avoid water vapor overpressure cooked under 500 W in a microwave for a specified time of 30, 60, and 120 s. The sample internal temperatures were measured immediately after cooking, and the mean values were 69, 74, and 81°C at 30, 60, and 120 s, respectively. All the cooking treatments were performed three times, and the samples were cooled to room temperature prior to analysis. The extraction process is described in Section 2.8.

### 2.8. Analyte Extraction Procedures

The analytical method used in this study for the determination of Amox in raw, cooked muscles and the surrounding fluids that remained after boiling were prepared, extracted, and analyzed by the previously reported method [24]. The method was revalidated for this work. Initially, pure Amox standard solution 100 mg L^−1^ was injected without cooking processes to obtain a maximum reference absorbance peak area value for the antibiotic. Thereafter the spiked, raw, cooked chicken samples and the surrounding fluids that remained after cooking were subjected to thermal stability test [25]. The drug residue stability was evaluated by comparing the residue concentration quantified in raw muscle with the concentration measured in the muscle after the different cooking procedures.

For analyte extraction, 4 g chicken tissue sample was taken in a 50 mL polypropylene centrifuge tube spiked with 100 mg L^−1^ Amox; the mixture was vortexed for 1 min, left to stand for 30 min to equilibrate, and homogenized using a blender for one minute; and the sample was divided into two portions. One portion (2 g) of the spiked raw sample was accurately weighed into a 25 mL polypropylene centrifuge tube, and the desired analyte was extracted by adding 10 mL acetonitrile, centrifuged at 3,000 rpm for 5 min. The upper organic extracted layer was filtered with a syringe filter and analyzed for raw analysis without cooking. The other spiked portions were subjected to different cooking procedures (boiling, frying, and microwave cooking) for various time intervals usually in household practice, and followed the similar procedure of extraction as the raw (uncooked) sample. Each eluted analyte was dried with a nitrogen stream produced through sample concentrator nitrogen. Then, the dried analyte was reconstituted with 2 mL of methanol and subjected to the LC system.

## 3. Results and Discussion

### 3.1. Stability of Amox Standards in Boiling Water and Cooking Oil

Before studying the effects of different cooking processes, the stability of Amox in boiling water and cooking oil was determined. Pure Amox was detected as a sharp peak at 4.186 min wherein no impurity was detected in the LC-UV chromatogram of the standard solution (Figure 2(a)). Exposure of the drug to chicken meat in boiled water or cooked oil at 100°C for 5–45 min caused it to degrade to four products. The chromatograms (Figures 2(b)–2(v)) show that the degradation of the Amox peak starts to split from the parent peak when the Amox was boiled for 5 min, and new peaks appeared after boiling for 15–30 min at 100°C, and 70 to 90% of the Amox degraded after 30 min boiling. Figures 2(i)–2(v) show the resulting chromatograms after boiling of Amox at different time intervals. It shows the main peak depletion Amox, and the resulted new peak appearance, and changes in the total peak area after heat treatment.

We have run blank of nonspiked chicken cooked under the same conditions and times. There was no interference peak observed before and after cooking as shown in Figures 3(a) and 3(b). However, after spiking the chicken tissue with Amox and cooking, new peaks appeared. This confirms the decomposition products of amoxicillin. But the structural changes, possible toxicity, and breakdown products were not studied and remained unclear [14].

### 3.2. The Effect of Boiling in Chicken Tissues

The cooking method for chicken meat in water at the boiling point of 100°C shows a statistically significant reduction of Amox concentration in the range of 70–87% after 30–45 min cooking (Table 1). The highest depletion of the residue may be the possibility of a loss of some Amox residues by leaching out from the cooked chicken muscle into the cooking medium or with juices [26]. The (supernatant) surrounding fluids in the boiling experiments detect 0.57 to 8.42% amounts of Amox residues. The residue concentration quantified for Amox did not show significant changes after boiling above 45 min cooking. A similar effect was observed for oxytetracycline in muscle [26]. The effects of cooking at 100°C by boiling the chicken tissue and muscle juice are represented in Figure 4.

### 3.3. Effect of Frying on the Residue Concentration

The frying process could help in reducing the Amox residues at 100°C for 5–30 min; the maximum reductions obtained were 25–92%. However, at 150°C for 30–45 min, the Amox concentration was increased. This might be due to dehydration or about 20% loss of water through evaporation from the meat sample during the cooking process [11]. A plot of amoxicillin concentration against time in hot oil is shown in Figure 5. At higher temperatures, i.e., 200°C, the peak of Amox has vanished, and only the degraded products remained; this result was agreed with the work of Svahn and Bjorklund [27]. Therefore, controlling the time and temperature of cooking is still needed to retain the taste and appearance of the food.

### 3.4. Effect of Microwaving in Chicken Tissues

The reduction of Amox in chicken tissue cooked by microwaving was rapid, and its residues were reduced by 0.03–11.06% in 0.5–2 min treatments.  Figure 6 shows the raw and cooked spiked tissue samples.

### 3.5. Degradation Percentage and Degradation Kinetics

Quantitative information about the depletion of the antibiotic residue by thermal treatment is mostly available in the literature through parameters such as degradation percentages or degradation rate constant (*k*) which is used to study the thermal kinetic of antibiotics [27–32]. The degradation kinetics of a chemical reaction, as a result of temperature, is defined by the Arrhenius equation, which relates the rate of a reaction increase with the increase in temperature [33]. From this kinetics parameter, the prediction models can be developed to estimate the concentration losses of antimicrobial compounds in terms of temperature and time. Roca and his coworkers [28] derived the predictive models to explain the thermal degradation of *β*-lactam antibiotic residues in milk by applying a first-order kinetic model and the Arrhenius equation from experimental time series and temperatures. The degradation percentages of Amox for different heat treatments were calculated according to

(1) $$\begin{array}{c} \text{degradation}\left(\%\right)=\frac{C_{0}-C_{f}}{C_{0}}\times 100, \end{array}$$

where C_0_ and *C*_*f*_ are the concentrations of the compounds before and after heat treatment, respectively [28]. The Amox degradation reaction rate was increased by increasing temperature since the kinetic constant raises with the temperature according to the Arrhenius law [33].

Ordinary cooking (forced degradation) procedures degrade the Amox residues depending on the amount of heat treatment and duration of heating involved [28]. A forced degradation study was subjected to check the stability of Amox in applied heat under stress conditions through boiling, frying, and microwave cooking methods. Amox showed variable stability for the different cooking processes of boiling, frying, and microwaving, as shown in Figure 7. The temperature and time effects on the depletion of Amox concentration were indicated in Table 1. Amox has high thermal stability and completely recovered at temperatures up to 150°C [27, 28]. The time factor (5, 30, and 45 min) showed a greater effect on the depletion of Amox compared to the temperature factor (100, 150, and 200°C). The results of the present study indicated that the Amox residue in chicken muscle shows a significant reduction (*p* < 0.05) for boiling procedures than microwave cooking. This may be due to the partially heat-labile nature of amoxicillin [27]. However, an increase in the concentration was observed in the pan-frying cooking process due to dehydration [14].

Table 1 summarizes the effect of different ordinary cooking methods on the concentration depletion of Amox residues in chicken tissue. The most reduced residue in cooked chicken samples is related to the boiling process, while the highest stable amount of residue belonged to microwave cooked samples. Regarding the results of this study, it could be concluded that cooking processes cannot annihilate the total amounts of this drug and it can only decrease its amounts. The initial findings from this investigation suggest that further work is needed to establish the behavior of Amox and its metabolites during cooking [34].

### 3.6. Validation

The analytical quality assurance of the method used for the analysis of residues of amoxicillin was validated by analyzing raw chicken muscle tissue samples spiked at three concentration levels 50, 100, and 200 *µ*g mL^−1^. The validation parameters were done based on the recommendations from ICH, 2005 guidance and evaluated for linear range, correlation coefficient (*R*^2^), recovery (%), precision (%), limit of detection (LOD), and limit of quantification (LOQ) [35].

The method linearity was investigated with six standard calibration points in the concentration range of 0.05 to 2 *µ*g mL^−1^. The calibration plots showed a linear relationship between the peak area responses versus the corresponding concentrations of the standard. The calibration plot linearity was in the concentration range of 0.05–250 *μ*g mL^−1^ with an acceptable correlation coefficient of 0.9994 as shown in Table 2. The limit of detection (LOD) and the limit of quantitation (LOQ) were 1.32 *µ*g mL^−1^ and 4.00 *µ*g mL^−1^, respectively, for the spiked raw chicken samples. Average sample recoveries (*n* = 6) were determined from negative control chicken tissue spiked at three concentration levels 50, 100, and 200 *µ*g mL^−1^ in raw samples. The obtained percentage recovery of Amox was between 78 and 106%. In the retention windows of the chromatograms of amoxicillin, no interferences were observed in the blank as well as in the spiked raw muscle samples. Repeatability (intraday precision) and reproducibility (interday precision) studies were conducted in order to evaluate the precision of the method and the corresponding maximum relative standard deviation RSD (%) values for all spiked levels were less than 8% that was complied with the requirement of the ICH, 2005 guidance which were lower than 20% [36].

### 3.7. Comparisons with Other Reported Literature Studies

In this method, cooking the chicken muscles by boiling brought significant reduction with varying percentages (Table 1). These results were in parallel with the findings reported by Vivienne and his coworkers [26], who recorded a significant reduction of boiling in oxytetracycline residue in experimentally induced bird muscles. In agreement with the currently presented amoxicillin results, oxytetracycline appears to be very heat labile, as it can be almost completely degraded during boiling in water for 30 min [26]. However, no clear trend was observed for direct comparison of degradation percentages and the effect of cooking in antimicrobials because the values reported in the literature vary widely depending on the type of treatment used, matrix, pH, time, and temperature.

## 4. Conclusion

This study has revealed that cooking processes induce partial destruction of antibiotic residues. The obtained results indicated that maximum depletion of Amox occurred at boiling and frying method of cooking followed by microwave cooking of broiler meat through efficient heat treatment of muscle tissue. Cooking time and temperature may play significant roles in antibiotic residue reduction while cooking food.

However, cooking processes cannot annihilate the total amounts of this drug, but it can only decrease the residue concentration in the boiling process. These drugs are excreted from tissue to cooking fluid during the boiling treatment. Cooking processes cannot be used as reliable methods to ensure the full-drug residue degradation but can contribute to a marked decrease in concentration. Although some veterinary drug residues are reduced and degraded by cooking processes, it is essential to perform toxicology experiments on the parent drug and metabolites of these drugs that are produced after cooking in order to monitor the potential adverse effects of drug residues on consumer health.

## Figures and Tables

**Figure 1:** Chemical structure of amoxicillin. The octanol-water partition coefficient (log K_ow_) _=_ 0.87, 0.97; acidity constant (pK_a_) _=_ 2.4, 2.8, 7.2 [22].

**Figure 2:** Chromatogram of Amox pure standard (100 *μ*g mL^−1^) before heat treatment (a); the consequent chromatograms after boiling (b), showing the splitting of the standard peak due to heat treatment or cooking (5 min); the main peak depletion of Amox, and the resulted quantifiable new peaks appeared after boiling the compound at 100°C (15–30 min) (c, d), and the changes in the total peak area after heat treatment by boiling for 45 min (e).

**Figure 3:** Chromatogram of blank of nonspiked chicken before (a) and after (b) cooking under the same conditions and times.

**Figure 4:** The effects of boiling on the depletion of Amox residue within different time periods from chicken tissue.

**Figure 5:** The effects of frying on the depletion of Amox residue within different temperatures and times from chicken tissue.

**Figure 6:** The effects of microwave cooking on the depletion of Amox residue within different temperatures and times from chicken tissue.

**Figure 7:** Temperature and time effects on the depletion of Amox concentration.

**Table 1:** The effect of various types of cooking processes on the concentration of Amox residues, in raw and cooked muscle samples.

	Cooking T (°C)	Cooking time (min)	New peaks (no.)	Conc. after cooking (*μ*g mL^−1^)	Degradation (%)	
Before heat treatment	Raw sample	—	—	—	99.94	—
A	Boiled Amox standard	100	30	2	97.45	2.55
F						
T	Fried Amox standard	100	15	4	72.65	27.35
E						
R	Boiled chicken tissue	100	5	2	99.42	0.58
			15	2	98.56	1.44
			30	4	29.82	70.18
H			45	4	12.28	87.72
E	Fluid from boiled muscle	100	5	2	4.61	4.61
A			15	2	6.85	6.85
T			30	4	8.42	8.42
			45	4	0.57	0.57
T	Fried chicken tissue	100	5	2	97.24	2.76
R			15	3	74.82	25.18
E			30	4	18.54	81.46
A			45	4	7.28	92.72
T		150	5	2	101.5	—
M			15	2	101.78	—
E			30	3	112.56	—
N			45	4	44.51	55.49
T		200	5	4	4.87	95.13
			15	4	0.84	99.16
			30	4	—	—
			45	4	—	—
	Microwaved chicken tissue	500 W	0.5	1	99.97	0.03
			1	2	89.86	10.14
			2	2	88.94	11.06

Initially, all raw and cooked samples were spiked with Amox standard (100 *μ*g mL^−1^).

**Table 2:** Characteristics of the analytical quality assurance for spiked chicken samples.

Description	Results
Calibration curve	*y* = 93109*x* + 12938
Linear range (*µ*g mL^−1^)	0.05–250
Correlation coefficient (*R*^2^)	0.9994
Mean recovery (%)	78.0–106.2
RSD (%)	≤8.32
LOD (*µ*g mL^−1^)	1.32
LOQ (*µ*g mL^−1^)	4.00
Repeatability (% RSD, *n* = 3)	4.8–7.2
Reproducibility (% RSD, *n* = 3)	5.2–8.1

## Data Availability

All the data are included in the manuscript.
